# Arm Movement Analysis Technology of Wushu Competition Image Based on Deep Learning

This article has been retracted.

**DOI:** 10.1155/2022/9866754

**Published:** 2022-08-12

**Authors:** Xiaoou Zhang, Xingdong Wu, Ling Song

**Affiliations:** ^1^Chinese Guoshu Academy, Chengdu Sports University, Chengdu 610041, China; ^2^School of Wushu, Chengdu Sports University, Chengdu 610041, China; ^3^Physical Education Department, Institute of Disaster Prevention, Langfang 065201, China; ^4^Physical Education Institute, Jimei University, Xiamen 361021, China

## Abstract

In order to improve the recognition accuracy of action poses for athletes in martial arts competitions, it is considered that a single frame pose does not have the temporal features required for sequential actions. Based on deep learning, this paper proposes an image arm movement analysis technology in martial arts competitions. The motion features of the arm are extracted from the bone sequence. Taking human bone motion information as temporal dynamic information, combined with RGB spatial features and depth map, the spatiotemporal features of arm motion data are formed. In this paper, we set up a slow frame rate channel and a fast frame rate channel to detect sequential motion of images. The deep learning model takes 16 frames from each video as samples. The softmax classifier is used to get the classification result of which action category the human action in the video belongs to. The test results show that the accuracy and recall rate of the arm motion analysis technology based on deep learning in martial arts competitions are 95.477% and 92.948%, respectively, with good motion analysis performance.

## 1. Introduction

As one of the national fitness sports, Wushu has a good mass foundation. Since the implementation of the national fitness plan outline, the number of people participating in sports activities has been increasing, and the content of mass sports activities has been rich and colorful. In order to meet people's sense of visual belonging and psychological expectations, the performance of the athlete's technical level will also change accordingly. Since the competitive martial arts competition was held, the competition rules have been continuously improved, which has put forward new requirements for coaches and athletes, requiring coaches and athletes to have the sensitivity to observe things and improve the level of scientific training. Computer vision involves more and more fields and has developed into an interdisciplinary field integrating digital image processing, machine learning, computer science, and other disciplines. In order to make the communication between computers and people smoother, researchers simulate the working principle of biological vision. This technology is used to analyze and recognize the input image information of martial arts human body so that the computer can better understand human language, posture, and other pieces of information and make corresponding feedback [1].

There are many pieces of sports video and image information in Wushu competition. Through these pieces of information, we can analyze various data of athletes or competitions. However, the amount of data is too large. If the method of manual analysis is used, it will greatly increase human and material resources. Therefore, intelligent action and behavior recognition are introduced. Therefore, obtaining and analyzing external information based on computer vision has become a research hotspot in recent years. As one of the important applications in human motion recognition, motion analysis is to track and analyze the human body in the video by establishing the geometric model of human motion and then study the behavior characteristics of human motion [2]. On the one hand, the function of image analysis of Wushu competition includes maintaining the competition order, creating a good competition atmosphere, and promoting the fairness, impartiality, and openness of competition results. On the other hand, it is to measure and evaluate the technical level of athletes and realize the macrocontrol of technical direction. In martial arts competitions, there are high requirements for athletes' action posture, and in some scenes with fierce sports, the residence time of most actions is very short, so it is very difficult for human eyes to judge the standard of actions. If the camera can be used to collect human actions, and the parameters such as joint point position and angle of human actions can be obtained through the processing of video frames, the actions can be analyzed and judged pertinently so as to provide more scientific guidance for athletes' training [3]. Based on deep learning, this paper studies the image arm movement analysis technology of Wushu competition. Through human movement recognition, it can provide some help for Wushu competition and training, reduce human investment, and improve the efficiency of Wushu training of athletes.

## 2. Arm Movement Analysis Technology of Wushu Competition Image Based on Deep Learning

### 2.1. Feature Extraction of Arm Movement in Wushu Competition

The arm movement of Wushu competition is the dynamic information that occurs in a period of time. The human bone sequence is composed of multiple frames of bone data at different times. Therefore, many research works take the bone frame as the constituent unit of the human bone sequence. However, the skeleton frame itself lacks the necessary dynamic information for action, so it is inappropriate to take the skeleton frame as an action unit. The goal of motion segmentation is to divide a continuous motion sequence into several meaningful continuous and nonoverlapping subsequences, and each subsequence is associated with an atomic motion unit or action [4–10]. In terms of motion segmentation based on 3D bone sequence, it mainly includes three ways: traditional clustering, temporal clustering, and supervised time series segmentation. Because action recognition is a supervised machine learning problem in most cases, the supervised time series segmentation algorithm is related to action recognition. The local representation of video is divided into two stages: spatiotemporal interest point detection and local description. Spatiotemporal point of interest detection does not need to eliminate the background first like the global representation but uses the statistical characteristics in the local feature description stage, so it can reduce the impact on the algorithm performance under the conditions of illumination, camera angle transformation, and occlusion [11]. In the process of Wushu training, taking the decomposition action as the unit, the complete action is gradually taught to the students. The decomposition action is not a static posture but an action segment with a short duration, including spatial posture information and local time motion information.

Motion recognition based on 3D bone sequence can be regarded as a classification problem of structured time series. Each frame bone represents a point in the multidimensional space, and the sequence formed by the evolution of bone frames with time is represented as the trajectory curve of the multidimensional space. Humans have different speeds when completing the same action due to individual differences, but their decomposition actions are almost the same [12]. Taking the martial arts action of raising and lowering the arm as an example, this action can be divided into six actions, including “nonraised arm,” “raised arm lower than the shoulder,” “raised arm higher than the shoulder,” “raised arm above the shoulder,” “raised arm below the shoulder,” and “fully lowered arm.” After detecting the spatiotemporal interest point in the video, the descriptor should be used to describe the point or region. According to the unique complexity of video data, the descriptor should be robust to the changes in video background, clutter, scale, and direction [13–21]. The so-called structure means that there are fixed topological constraints between the joint positions of bones in each frame; for example, the head joint is only connected with the neck joint. Equivalently, there are numerical constraints between the coordinates of each joint [22]. Inspired by this, we define an action unit as a decomposition action that lasts for a short period of time. In the bone sequence, the action unit is defined as a bone fragment composed of several consecutive bone frames with similar spatial structure. A sequence of bones containing *N* frames of bones can be expressed as

(1) $$\begin{array}{c} w\left(N\right)=\left[a\left(N\right),b\left(N\right),c\left(N\right)\right]. \end{array}$$

In formula (1), *w*(*N*) represents the bone sequence. *N* represents the number of sequence frames. *a*(*N*), *b*(*N*), *c*(*N*) are the coordinate of the joint. When a person performs an action in the scene, the position of his arm changes every time. To eliminate this effect, translate the skeleton from a Kinect-centered coordinate system to a human-centered coordinate system for each frame. The coordinates of joints are related to the total number of joint points in the bone model. This paper mainly uses the bone model with a total number of joint points of 20. In order to reduce the sensitivity of the bone sequence to the shooting angle, the original bone sequence needs to be transformed into a reference coordinate system determined by the bone sequence itself [23]. The value of the new coordinate system origin can be expressed as

(2) $$\begin{array}{c} O=-\frac{\sum_{N=1}^{n}w_{1}\left(N\right)}{N}. \end{array}$$

In formula (2), *O* represents the origin value of the bone sequence coordinate system and *w*_1_(*N*) represents the center of the arm joint. The plane composed of joint points in the arm set is similar to the frontal plane, which divides the human body into front and back parts along the left and right diameters of the body. After the spatiotemporal interest point in the image is detected, the descriptor should be used to describe the point or region [24]. In view of the unique complexity of Wushu competition image data, the descriptor should be robust to video background, clutter, scale, and direction changes.

### 2.2. Spatiotemporal Feature Fusion of Arm Motion Data

The action behavior of the human body not only has discrimination in image space but also has discrimination in time series. Image recognition, detection, and other tasks need to mine spatial features, while video increases the information of time dimension relative to image. Therefore, a human motion recognition algorithm needs to deeply mine its temporal and spatial features. The commonly used multimodal information includes image static information, scene depth information, human bone point motion information, video sound information, and so on. The normalized bone sequence is automatically divided into multiple bone segments, and then the spatial and local time-domain features of bone segments are extracted and clustered to form a key segment dictionary [25]. The bone segment in the bone sequence is replaced by the key segment closest to it in the key segment dictionary. In this way, the bone sequence is encoded as a word sequence. Hierarchical representation is widely used in the field of computer vision, rather than just static motion recognition. Hierarchical representation is a strategy based on different particle size division to realize the recombination of spatiotemporal features. Static information is mainly aimed at space, including the global information about environment and human body. In static action recognition, the purpose of hierarchical representation is to consider the spatial layout of human-object interaction. If the spatial layout of human-object interaction in the image is not considered at all, there is basically no difference between static action recognition and object recognition. Hierarchical representation has become the most popular way of modeling human-object spatial relationship in the second kind of methods.

The static information used in this paper is RGB (Red, Green, Blue) map and depth map. RGB map contains the global information of environment and human body, and depth map reflects the more accurate position information of object and human body, which can be used to eliminate the problem of background mixing. Compared with static information, dynamic information increases the description of time dimension. This paper uses human bone motion information as dynamic information. It is not enough to only obtain the absolute position information of each bone key point in the picture as human characteristics. It is also necessary to analyze the mutual position relationship between each bone key point to obtain the relative information between each joint point. For videos with multimodal information, both RGB and depth maps can mine spatial features, and RGB features can better express the color, texture, and other features of the human body or background in the video. The depth of the human body can be distinguished from the background. This paper uses RGB images to represent the color and texture features of the human body and background in videos. The CNN (Convolution Neural Network) used for depth images can accurately distinguish the front and back scenes of the video and prevent the wrong feature understanding caused by background interference. Feature points are set at the corresponding vertex position of each part, which constitute the star graph of human posture. Finally, the motion vector formed by the star graph is used as the feature vector to judge human action. The spatial depth feature can be expressed as

(3) $$\begin{array}{c} G=\frac{\alpha_{1}}{\alpha_{1}+\alpha_{2}}\beta_{1}+\frac{\alpha_{2}}{\alpha_{1}+\alpha_{2}}\beta_{2}. \end{array}$$

In formula (3), *G* is the output probability of spatial depth characteristics; *α*_1_ and *α*_2_ are the accuracy of the model; and *β*_1_ and *β*_2_ represent RGB map and depth map features. Human actions in video have temporal characteristics, so only mining spatial depth characteristics cannot express the temporal characteristics of actions. In the task of human motion recognition, the trajectory of human key bone points has effective time information. RNN (Recurrent Neural Network) model is a special neural network structure, which is based on the view that “human cognition is based on past experience and memory.” It not only considers the input of the previous moment but also endows the network with a “memory” function of the previous content. The model is good at solving sequence problems, where the discrimination and prediction of input data are related to adjacent data. It is suitable for solving the problem of martial arts action video sequences. This paper obtains the time characteristics of behavior by learning the trajectory of bone points. According to the two-dimensional distribution map of human bone key points, it can be found that three adjacent bone key points will form two adjacent limbs, and the included angle between two adjacent limbs can be calculated according to the cosine theorem. This series of angles can form a sequence, which can be used as the feature vector representing the human body. The final fusion result can be expressed as

(4) $$\begin{array}{c} F=\frac{1}{m}\left(\sum_{m=1}^{n}\vartheta G+\left(1-\vartheta \right)H\right). \end{array}$$

In formula (4), *F* represents the feature fusion result. *m* is the number of sample features after multiple sampling of Wushu competition video. *ϑ* is the weighting parameter. *H* represents the output probability of the time depth characteristic network. Based on these pieces of multimodal information, the spatiotemporal depth feature of this paper can improve the recognition accuracy by mining the characteristics of temporal and spatial information of actions.

### 2.3. Sequential Action Detection of Wushu Competition Images

The task of sequential action detection is to determine the time interval (including start time and end time) and the category of action in the video sequence. Because there are many kinds of movements in Wushu competition, including not only a single movement but also many complex movements composed of simple movements and the interaction between people and other auxiliary objects, it constitutes the complexity of movements. Single frame pose does not have the time characteristics necessary for sequential action, so it affects the accuracy of action recognition. Generally, the characteristics of one-dimensional time signals, such as acceleration, can be divided into time-domain characteristics, frequency-domain characteristics, and time-frequency-domain characteristics [26]. The features extracted from different dimensions have a great impact on the final classification results. Here, we use the fast Fourier transform coefficients as the representation of frequency-domain features. In the process of detection, it mainly depends on the identification of action key frames, which are mainly the start frame, action change frame, and end frame. The key task of key frame recognition is to start and end an action and test whether the action is standardized at the node of the key frame. The so-called time-frequency characteristics are generally based on wavelet analysis. Wavelet analysis can not only reflect the frequency-domain characteristics of data but also reflect the time-domain characteristics of data. In the network structure of this paper, a slow frame rate channel and a fast frame rate channel are set. In the slow frame rate channel, the network has a low refresh speed in order to obtain the spatial information in the video frame. In another fast frame rate channel, refresh quickly at a higher frame rate and obtain the rapid change of action at a higher time resolution.

By connecting the convolution between high resolution and low resolution in parallel, the network has been in high-resolution representation. In order to enhance this high-resolution representation, the network not only uses the common method of recovering high-resolution representation from low-resolution representation but also combines repeated cross-parallel convolution to perform multiscale fusion of features. Many researchers have studied the recognition task based on wavelet analysis. Here, we use wavelet packet decomposition (WPD) as the feature extraction method of acceleration signal. When calculating the FFT coefficients of the segmented data, the fast Fourier transform is performed on the *x*-axis, *y*-axis, and *z*-axis, respectively. Here, taking the *x*-axis as an example, the transformed 2nd- to 64th-bit data are taken as the final FFT coefficients. The timing detection model is mainly composed of three parts: feature extraction subnet, timing detection subnet, and action classification subnet, as shown in Figure 1.

The output decomposition structure consists of wavelet decomposition vector and bookkeeping vector, which contains coefficients divided by level. Like the operation mode of FFT coefficients, WPD features are extracted from the segmented three-axis acceleration data through the above functions, and then the three-axis data are sorted into a one-dimensional feature representation. The combination of the two makes the whole network not only maintain high-resolution information but also integrate low-resolution information, which significantly improves the effect of keypoint detection.

The goal of the fast frame rate channel is to obtain the description of actions in video in time dimension. There are three requirements for the setting of a fast frame rate channel: first, it has a large frame rate, which can obtain the motion information of action; second, it has higher resolution. In order to obtain higher resolution, no pooling layer is used in the whole fast frame rate channel; that is, the resolution of the input video frame remains unchanged; third, the occupied channel capacity is small. Here, the channel capacity is set to be 1/8 of the channel capacity of slow frame rate, which will also bring small calculation and reduce the amount of calculation. Generally speaking, the network is composed of four parallel subnets, including four stages. In the first stage, the high-resolution subnet is used, then in each stage, the resolution is reduced to 1/2 of the original, and the width (the number of channels) is doubled. In the last stage, the fused highest resolution is used to recognize the arm movement in Wushu competition.

### 2.4. Establishment of the Arm Motion Analysis Model Based on Deep Learning

In the analysis of arm movement in Wushu competition images, the processed data are no longer a single image but an image sequence with time sequence. If each frame in the video is treated as input data, the computational cost of the model will be greatly increased. It can be seen from the definition of progress label that progress label is related to the action category. A network can only learn the progress label information of one kind of action [27]. Therefore, it is necessary to train the progress label prediction network belonging to each kind of action *k*. The training data are the video frame of the action instance belonging to the *k*-th progressive action in the training video sample. Therefore, the depth learning model in this paper takes 16 frames from each video as samples. Then, input the samples into the model to learn the network weight. Finally, the softmax classifier is used to complete the action recognition. In machine learning, especially deep learning, softmax is a very common and important function, especially in multiclassification scenarios. He maps some inputs to real numbers between 0 and 1, and the normalization guarantees that the sum is 1, so the sum of the probabilities of multiclassification is also exactly 1. This model is useful for problems such as human action classification.

The overall architecture of the model includes three parts: data processing, feature extraction, and action recognition. The overall architecture of the model also includes two full connection layers. The training data can only be the video frames in the progressive action instance because if the video frames in the nonprogressive action instance are added to the training, it will bring noise, confuse the training objectives, and weaken the learning ability of the network. The function of the first FC layer is to integrate the previously extracted spatial features and then send them to the network of the next layer for learning. The function of the second FC layer is to map the final output feature of the model to the label space of the action sample through linear transformation [28]. The loss function is defined as the average absolute error between the predicted value and the true value, as shown in

(5) $$\begin{array}{c} f=\frac{\sum_{n=1}^{u}n\left|\lambda -\gamma \right|}{u}. \end{array}$$

In formula (5), *f* represents the loss function; *u* is the total number of frames of training samples; *λ* and *γ* are the predicted value and true value of the *i*-th frame image sample, respectively. Because the original resolution of video data is usually large and the calculation cost of direct use is high, it needs to be preprocessed. The traditional data preprocessing process is as follows. The video is parsed into video frame sequence by the ffmpeg module, and the original video frame is scaled according to the training requirements. The scaled video frame is recropped, the cropped video frame is transformed into tensor form, and finally, the tensor is regularized. In addition to two convolution layers and a residual connection, each residual block also includes a lightweight multiscale convolution module and channel attention mechanism [29]. Then, after successfully passing through the flatten layer (compressing the information of the feature map in all dimensions to one dimension), the FC layer, and the softmax classification layer, the classification result of which action category the human action in the video belongs to is finally obtained. Compared with the ordinary network, the residual network adds a shortcut connection on its basis. Therefore, the output result of the residual module is

(6) $$\begin{array}{c} Y\left(\varphi \right)=Z\left(\varphi \right)+\varphi . \end{array}$$

In formula (6), *Y*(*φ*) represents the output result of the residual module; *Z*(*φ*) represents the output result of shortcut connection; *φ* indicates the input target. If the shallow network has reached the accuracy of saturation, by adding several identity mapping layers behind it, the purpose of increasing the network depth without increasing the training error can be realized; that is, the degradation problem of deep network can be solved. All convolution layers are followed by batch normalization operation and ReLU activation function. Among them, the BN operation makes the output specification after convolution equal to 0 and the variance equal to 1, which can basically eliminate the disappearance of the backpropagation gradient and accelerate the convergence speed of the model [30]. The nonlinear output can be obtained by using the ReLU activation function, and the problem of gradient dispersion can be alleviated to a certain extent. So far, the research on martial arts movement based on image analysis is completed.

## 3. Experiment

### 3.1. Experimental Preparation

In this experiment, the arm movement dataset of Wushu competition is established. Based on the collected data samples, the image arm movement analysis technology of Wushu competition based on deep learning is tested. Collect the competition videos of the top 5 athletes of men's group, a self-selected Taijiquan and Taijijian, the top 5 athletes of women's group, a self-selected Taijiquan and Taijijian, and the top 10 athletes of men's and women's self-selected Taijiquan and Jian in the National Wushu routine championship. The database contains 256 video sample data, and the average number of frames contained in the video is 6792. In the effective video samples in the database, there are 498 target actions to be detected, and the average number of frames contained in the target actions to be detected is 2473 frames. The martial arts arm movements selected in this experiment are two arms straightening, two arms forced backward and upward vibration, and two arms circling. The number of target movements to be detected in the above three movements are 258, 247, and 268, respectively. The arm movement dataset used in the experiment is divided into 60% as a training set, 20% as a verification set, and 20% as a test set. In order to reduce the occurrence of overfitting, the size of the final input video stream is 128^*∗*^171^*∗*^3^*∗*^16, which corresponds to the length, width, number of channels, and length of the video frame, respectively. The network uses a total of 8 convolution layers, 5 maximum pooling layers, and 2 fully connected layers. Finally, softmax is connected as the output layer. The convolution kernel size ranges from 64 in the lower layer to 512 in the upper layer, and the corresponding feature expression is also a process from general to special. The training adopts the random gradient descent method to update the weight, and the learning rate is initially set to 0.01. The deep learning development environment used in this paper is Anaconda + Pycharm, and the programming language is Python.

### 3.2. Experimental Results and Analysis

In order to test the performance of the image arm motion analysis technology of Wushu competition based on deep learning, the recognition accuracy and recall rate are selected as the evaluation indexes to evaluate the motion analysis technology. The experimental results of arm motion analysis technology in this paper are compared with the image arm motion analysis technology of Wushu competition based on SVM and LSTM. The analysis results of arm movement are shown in Figures 2–4.

From the above test results, it can be seen that the method proposed in this paper can accurately identify the joint points of Wushu arm movement, and users can intuitively see their key posture during movement training. In the subsequent training process, users can make targeted adjustments to maintain the more standard actions and improve the actions that are not standard so as to make their training actions closer and closer to the standard template actions and improve the overall training effect. This paper extracts the motion features of the arm through the bone sequence. The human bone motion information is used as the time dynamic information. It combines the spatial features of RGB and the depth map to form the spatiotemporal features of the arm motion data. This paper can more accurately identify martial arts arm movements. There is a large deviation in the joint point positioning of the other two comparison schemes. The comparison results of recognition accuracy and recall are shown in Tables 1 and 2, respectively.

According to the test results in Table 1, the recognition accuracy of the martial arts competition image arm movement analysis technology based on deep learning is 95.477%, which is 5.296% and 3.174% higher than that of the martial arts competition image arm movement analysis technology based on SVM and LSTM, respectively.

According to the test results in Table 2, the recall rate of martial arts competition image arm movement analysis technology based on deep learning is 92.948%, which is 7.039% and 5.808% higher than that of martial arts competition image arm movement analysis technology based on SVM and LSTM, respectively.

Due to the use of different modes in the video and different network structures and classifiers, all fusion adopts the method of linear fusion. By embedding a lightweight multiscale convolution module into the convolution residual network, the receptive field size of each convolution layer is greatly increased, so a better classification effect can be achieved. The experimental results show that deep learning obtains better results based on a large number of training data. The action description of the image arm action analysis technology of Wushu competition proposed in this paper is interpretable, which is convenient to analyze the internal situation of the action, and can improve the accuracy of action classification.

## 4. Conclusion

1. This paper studies the arm movement analysis technology of martial arts competition images based on deep learning. The motion features of the arm are extracted from the bone sequence. Taking human bone motion information as temporal dynamic information, combined with RGB spatial features and depth map, the spatiotemporal features of arm motion data are formed. The deep learning model takes 16 frames from each video as samples, learns the network weights, and uses the softmax classifier to get the classification result of which action category the human action in the video belongs to. The experimental results show that the technology can improve the accuracy and recall rate of arm action recognition and is suitable for the analysis of related modal information of similar videos. The test results show that the accuracy and recall rate of the arm motion analysis technology based on deep learning in martial arts competitions are 95.477% and 92.948%.
2. Since most of the human action recognition datasets come from the sharing of video websites or video footage, there is a lot of noise in the data, so how to effectively reduce the noise of the video is also a future research work worthy of further exploration. Most videos on the web contain not only action sequences but also other pieces of irrelevant information. Therefore, in practical applications, actions need to be detected first and then recognized.
3. At present, this method cannot provide the function of motion detection, which undoubtedly increases the difficulty of practical application. Therefore, it is necessary to combine the action detection method in the video with this method to realize the video action recognition function of any video [31].

## Figures and Tables

**Figure 1:** Sequence detection process.

**Figure 2:** Analysis technology of image arm movement in Wushu competition based on deep learning. (a) Preparation action. (b) Block. (c) Hook fist. (d) Straight fist.

**Figure 3:** Analysis technology of image arm movement in Wushu competition based on SVM. (a) Preparation action. (b) Block. (c) Hook fist. (d) Straight fist.

**Figure 4:** Analysis technology of image arm movement in Wushu competition based on LSTM. (a) Preparation action. (b) Block. (c) Hook fist. (d) Straight fist.

**Table 1:** Comparison of accuracy (%).

Number of tests	Arm movement analysis technology of Wushu competition image based on deep learning	Arm movement analysis technology of Wushu competition image based on SVM	Arm movement analysis technology of Wushu competition image based on LSTM
1	94.464	90.106	91.486
2	95.838	91.458	92.817
3	96.606	90.884	91.561
4	94.323	89.561	92.634
5	95.252	90.630	92.354
6	96.515	90.222	91.228
7	95.171	89.535	92.519
8	94.484	88.199	93.146
9	96.852	90.472	92.472
10	95.263	90.743	92.808

**Table 2:** Comparison of recall rate (%).

Number of tests	Arm movement analysis technology of Wushu competition image based on deep learning	Arm movement analysis technology of Wushu competition image based on SVM	Arm movement analysis technology of Wushu competition image based on LSTM
1	93.106	87.475	88.449
2	94.468	86.886	89.185
3	91.824	85.547	88.567
4	92.527	86.114	86.834
5	93.611	84.261	87.651
6	92.375	85.638	86.378
7	91.082	86.352	88.016
8	92.223	85.026	85.243
9	93.506	86.279	84.782
10	94.759	85.512	86.295

## Data Availability

The data used to support the findings of this study are available from the corresponding author upon request.
